The article "Pravastatin Attenuates Acute Radiation-Induced Enteropathy and Improves Epithelial Cell Function" was published in 2018. Journal: Front Pharmacol.

# Pravastatin Attenuates Acute Radiation-Induced Enteropathy and Improves Epithelial Cell Function

**DOI:** 10.3389/fphar.2018.01215

**Published:** 2018-10-30

**Authors:** Hyosun Jang, Janet Lee, Sunhoo Park, Hyunwook Myung, Jihoon Kang, Kyuchang Kim, Hyewon Kim, Won-Suk Jang, Sun-Joo Lee, Sehwan Shim, Jae K. Myung

**Affiliations:** ^1^Laboratory of Radiation Exposure & Therapeutics, National Radiation Emergency Medical Center, Korea Institute of Radiological and Medical Sciences, Seoul, South Korea; ^2^Department of Pathology, Korea Cancer Center Hospital, Korea Institute of Radiological and Medical Sciences, Seoul, South Korea

**Keywords:** pravastatin, radiation-induced enteropathy, intestinal epithelial cells, oxidative stress, irradiation

## Abstract

**Background and Aim:** Radiation-induced enteropathy is frequently observed after radiation therapy for abdominal and pelvic cancer or occurs secondary to accidental radiation exposure. The acute effects of irradiation on the intestine might be attributed to inhibition of mitosis in the crypts, as the loss of proliferative functions impairs development of the small intestinal epithelium and its barrier function. Especially, oxidative damage to intestinal epithelial cells is a key event in the initiation and progression of radiation-induced enteropathy. Pravastatin is widely used clinically to lower serum cholesterol levels and has been reported to have anti-inflammatory effects on endothelial cells. Here, we investigated the therapeutic effects of pravastatin on damaged epithelial cells after radiation-induced enteritis using *in vitro* and *in vivo* systems.

**Materials and Methods:** To evaluate the effects of pravastatin on intestinal epithelial cells, we analyzed proliferation and senescence, oxidative damage, and inflammatory cytokine expression in an irradiated human intestinal epithelial cell line (InEpC). In addition, to investigate the therapeutic effects of pravastatin in mice, we performed histological analysis, bacterial translocation assays, and intestinal permeability assays, and also assessed inflammatory cytokine expression, using a radiation-induced enteropathy model.

**Results:** Histological damage such as shortening of villi length and impaired intestinal crypt function was observed in whole abdominal-irradiated mice. However, damage was attenuated in pravastatin-treated animals, in which normalization of intestinal epithelial cell differentiation was also observed. Using *in vitro* and *in vivo* systems, we also showed that pravastatin improves the proliferative properties of intestinal epithelial cells and decreases radiation-induced oxidative damage to the intestine. In addition, pravastatin inhibited levels of epithelial-derived inflammatory cytokines including IL-6, IL-1β, and TNF-α in irradiated InEpC cells. We also determined that pravastatin could rescue intestinal barrier dysfunction via anti-inflammatory effects using the mouse model.

The article "Pravastatin Attenuates Acute Radiation-Induced Enteropathy and Improves Epithelial Cell Function" was published in 2018. Journal: Front Pharmacol.

**Conclusion:** Pravastatin has a therapeutic effect on intestinal lesions and attenuates radiation-induced epithelial damage by suppressing oxidative stress and the inflammatory response.

## Introduction

As the intestine is highly sensitive to ionizing radiation, radiation-induced enteropathy is frequently observed radiation therapy for abdominal or pelvic cancers including gastric, pancreatic, and endometrial cancer or can occur secondary to accidental radiation exposure (Kavanagh et al., 2010). Radiation-induced enteritis is associated with a defined pattern of acute inflammation and chronic fibrosis that is induced by a series of processes including ROS production, DNA damage, lipid peroxidation, and apoptosis. The acute effects of irradiation on the intestine can be attributed to inhibition of mitosis in the crypts; moreover, the loss of proliferative function impairs the development of the small intestinal epithelium and increases intestinal permeability, which results in increased translocation of luminal bacteria into the systemic compartment, generating a local and systemic immune response (Son et al., 2013; Yu, 2013). Whereas these issues have prompted increased interest in the development of therapeutic agents for radiation enteropathy in cancer patients and victims of radiation disasters (Potten, 1990; Pritchard et al., 1999; Greenberger, 2009; Citrin et al., 2010), there are no FDA-approved agents for the prevention or treatment of this disease (Greenberger, 2009; Citrin et al., 2010; Yu, 2013).

Radiation injury is mainly caused by the overproduction of ROS, which are products of the respiratory chain in mitochondria (Yamamori et al., 2012), a damaged anti-oxidant system, or a combination of these issues. Oxidative stress leads to the suppression of cell proliferation and increases in apoptosis and DNA damage (Jacobson, 1996; Keates et al., 1997; Ding et al., 2007). Especially, oxidative stress-induced damage to intestinal epithelial cells is a key event in the initiation and progression of radiation-induced enteropathy pathologies (Jeong et al., 2016; Abd El-Hady et al., 2017). Because differentiated epithelial cells of the small intestine are involved in fluid and nutrient absorption, oxidative damage to epithelial cells through radiation exposure leads to a malabsorptive state in which unabsorbed nutrients, electrolytes, and water are deposited into the distal segments of the gastrointestinal tract, resulting in nausea, vomiting, and diarrhea. Therefore, the reduction of oxidative stress to intestinal epithelial cells is responsible for recovery from acute irradiation effects.

3-Hydroxy-3-methylglutaryl coenzyme A (HMG-CoA) reductase inhibitors, also known as statins, are widely used in the clinic to lower serum cholesterol and were reported to have therapeutic applications for a range of inflammatory conditions (Rosenson, 1999; Nakamura et al., 2006). Moreover, statins have beneficial effects on radiation-induced toxicities, and numerous studies have demonstrated the anti-inflammatory effects of pravastatin, which occurs through improved endothelial cell function following radiation exposure (Gaugler et al., 2005; Haydont et al., 2007; Holler et al., 2009). However, there are limited reports regarding the effects of statins on intestinal epithelial cells damaged by radiation.

The article "Pravastatin Attenuates Acute Radiation-Induced Enteropathy and Improves Epithelial Cell Function" was published in 2018. Journal: Front Pharmacol.

In this study, we investigated the therapeutic effects of pravastatin on the acute radiation-induced enteropathy, focusing on intestinal epithelial cells. We showed that intestinal epithelial cells exhibit reduced proliferative ability in response to radiation toxicity, but that pravastatin treatment attenuates intestinal epithelial cell damage. Down-regulation of oxidative stress by pravastatin results in a diminished inflammatory response and the recovery of epithelial barrier dysfunction. Pravastatin showed therapeutic effects against acute radiation-induced enteropathy in mice. These results suggest that pravastatin is effective against acute radiation-induced enteritis through the upregulation of proliferation and anti-oxidative functions in intestinal epithelial cells, thus attenuating inflammation and improving intestinal barrier function.

## Materials and Methods

### Mice

Specific pathogen-free (SPF) male C57BL/6 mice (7-week-old) were obtained from Harlan Laboratories (Indianapolis, IN, United States) and maintained under SPF conditions at the animal facility of the Korea Institute of Radiological and Medical Sciences (KIRAMS). All mice were housed in a temperature-controlled room with a 12-h light/dark cycle, and food and water were provided *ad libitum*. The mice were acclimated for 1 week before experiments and assigned to the following groups: (1) control (*n* = 25), (2) irradiation (IR, *n* = 25), and (3) irradiation with pravastatin treatment (IR + Prava, *n* = 25). All animal experiments were performed in accordance with the guidelines of and were approved by the Institutional Animal Care and Use Committee of KIRAMS.

### Irradiation and Administration of Pravastatin

Animals were anesthetized with an intraperitoneal injection of 85 mg/kg alfaxalone (Alfaxan^®^; Careside, Gyeonggi-do, South Korea) and 10 mg/kg xylazine (Rompun^®^; Bayer Korea, Seoul, South Korea). They were then irradiated with a single exposure to 13.5 Gy of whole abdominal irradiation at a dose rate of 2 Gy/min using an X-RAD 320 X-ray irradiator (Softex, Gyeonggi-do, South Korea). After exposure, animals were treated with a daily oral dose of 30 mg/kg/day pravastatin (Prastan^®^; Yungin Pharm, Seoul, South Korea) for 6 days.

The article "Pravastatin Attenuates Acute Radiation-Induced Enteropathy and Improves Epithelial Cell Function" was published in 2018. Journal: Front Pharmacol.

### Histological Analysis of the Intestine

Small intestine samples of mice were fixed with a 10% neutral buffered formalin solution, embedded in paraffin wax, and sectioned transversely to a thickness of 4 μm. The sections were then stained with hematoxylin and eosin (H&E). To perform immunohistochemical analysis, slides were performed heat-induced antigen retrieval in Tris-EDTA pH9 buffer and then treated with 0.3% hydrogen peroxide in methyl alcohol for 20 min to block endogenous peroxidase activity. After three washes in PBS, the sections were blocked with 10% normal goat serum (Vector ABC Elite kit; Vector Laboratories, Burlingame, CA, United States) and incubated with anti-mucin 2 (Muc2; Abcam, Cambridge, United Kingdom), anti-lysozyme 1 (Lyz1; Abcam), anti-chromogranin A (ChgA; Abcam), anti-Ki-67 (Acris), anti-8-hydroxy-2′-deoxyguanosine (8-OHdG; Abcam), anti-myeloperoxidase (MPO; Abcam), and claudin 3 (CLDN3; Invitrogen, Carlsbad, CA, United States) antibodies. After three washes in PBS, the sections were incubated with a horseradish peroxidase-conjugated secondary antibody (Dako, Carpinteria, CA, United States) for 60 min. The peroxidase reaction was developed using a diaminobenzidine substrate (Dako) prepared according to the manufacturer’s instructions, and the slides were counterstained with hematoxylin. Apoptotic cell death was assessed using a terminal deoxynucleotidyl transferase dUTP nick and labeling (TUNEL) assay (Sigma-Aldrich, St. Louis, MO, United States).

### Cell Culture

The InEpC normal human intestinal epithelial cell line was purchased from Lonza (Walkersville, MD, United States) and were grown in SmBM medium containing supplements (SmBM-2 BulletKit, Lonza) at 37°C in a humidified atmosphere containing 5% CO_2_. Cells were irradiated with 13 Gy of irradiation using a ^137^Cs γ-ray source (Atomic Energy of Canada, Chalk River, ON, Canada) at a dose rate of 3.81 Gy/min and then treated with pravastatin (Sigma-Aldrich, St. Louis, MO, United States) within 1 h. After 48 h of incubation, the cells were used for experiments.

### Proliferation Assays

Cell proliferation was evaluated using a colorimetric method based on WST-1 (CellVia, Abfrontier, Seoul, South Korea). Next, 5 × 10^3^ cells were seeded in 96-well culture plates. Cells were irradiated and then treated with various doses of pravastatin. After a 48-h incubation, 10 μL of CellVia was added and the cells, which were incubated for an additional 1 h at 37°C. Proliferation was measured using a microplate reader at a wavelength of 450 nm.

The article "Pravastatin Attenuates Acute Radiation-Induced Enteropathy and Improves Epithelial Cell Function" was published in 2018. Journal: Front Pharmacol.

### Senescence-Associated β-Galactosidase (SA β-Gal) Staining

Cells were fixed with 4% formaldehyde and stained for β-gal activity using a Senescence β-Gal Staining Kit (Cell Signaling, Danvers, MA, United States). Positive cells were counted from three random fields for each group, and total cell number was also determined.

### Mitochondria Superoxide and Cellular ROS Assays

Mitochondrial superoxide generation was detected after staining cells for 10 min at 37°C with 5 μM MitoSOX Red (Invitrogen), a mitochondrial superoxide indicator, and DAPI for nuclear staining. Cells were then washed with PBS before imaging. To determine cellular ROS levels, cells were incubated with 10 nM 2′,7′-dichlorofluorescein diacetate (DCF-DA; Molecular Probes, Inc., Eugene, OR, United States). The cells were then harvested by trypsinization and analyzed for DCF-DA fluorescence using fluorescence-activated cell sorter analysis. Groups of cells were randomly selected from each sample.

### Glutathione (GSH) Assays

Cellular GSH was measured spectrofluorometrically using a GSH Colorimetric Detection Kit (Biovision, Milpitas, CA, United States). Cell pellets were lysed in 100 μL of ice-cold cell lysis buffer. They were then incubated on ice for 10 min and centrifuged for 10 min, and the cell lysate was transferred for GSH assays. The reactions were incubated at 37°C for 30 min, and values were measured using a multi microreader at an excitation/emission of 380/460 nm.

### RNA Extraction, Reverse Transcription-Polymerase Chain Reaction (RT–PCR), and Real-Time PCR Quantification

Harvested mouse small intestine tissues were immediately snap-frozen and stored at -80°C until RNA extraction. Total RNA was isolated from the intestine tissues using the TRIzol reagent (Invitrogen, Carlsbad, CA, United States), and total RNA from InEpC cells was extracted using the RNeasy mini kit (Qiagen, Hilden, Germany). cDNA was synthesized using the AccuPower RT premix (Bioneer, Daejeon, South Korea) according to the manufacturer’s protocol. Real-time RT-PCR was performed using a LightCycler 480 system (Roche, San Francisco, CA, United States). The primer sequences are provided in Table 1. The expression levels of each target gene, determined using the LightCycler 480 system software (Roche), were normalized to those of β-actin. Cycle threshold values were used to calculate relative mRNA expression using the 2^-ΔΔCt^ method.

The article "Pravastatin Attenuates Acute Radiation-Induced Enteropathy and Improves Epithelial Cell Function" was published in 2018. Journal: Front Pharmacol.

**Table 1:** Real-time RT-PCR primer sequences.

Species	Primer	Forward (5′–3′)	Reverse (5′–3′)	bp
Human	TNF-α	CAGAGGGCCTGTACCTCATC	GGAAGACCCCTCCCAGATAG	219
	IL-1β	AATCTGTACCTGTCCTGCGTGTT	TGGGTAATTTTTGGGATCTACACTCT	78
	IL-6	TGAGAGTAGTGAGGAACAAG	CGCAGAATGAGATGAGTTG	189
	GAPDH	GGACTCATGACCACAGTCCATGCC	TCAGGGATGACCTTGCCCACAG	152
Mouse	Il-1β	GGTCAAAGGTTTGGAAGCAG	TGTGAAATGCCACCTTTTGA	94
	Tnf-α	GCCTCTTCTCATTCCTGCTT	CACTTGGTGGTTTGCTACGA	203
	Mmp-9	GCCCTGGAACTCACACGACA	TTGGAAACTCACACGCCAGAAG	85
	Cldn 3	AAGCCGAATGGACAAAGAA	CTGGCAAGTAGCTGCAGTG	72
	β-Actin	TCCCTGGAGAAGAGCTATGA	CGATAAAGGAAGGCTGGAA	100

### Bacterial Translocation Assays

To evaluate the translocation of bacteria, from the intestinal lumen to lymph nodes, mLNs of mice were harvested under sterile conditions 6 days following IR. An aliquot of the mLN homogenate was plated onto MacConkey agar (BD, Franklin Lakes, NJ, United States) and incubated at 37°C for 18 h. Then, colonies were counted on all plates.

### Intestinal Permeability Assays

Animals were anesthetized and a midline laparotomy was performed. A 5-cm segment of digital ileum was obstructed using bulldog clamps. An intraluminal injection of 12.5 mg FITC-dextran (4 kDa, Sigma, St. Louis, MO, United States) in 100 μL PBS was the performed at 3 and 6 days following IR. At 30 min following intraluminal injection, blood was obtained via cardiac puncture and placed in serum-separating tubes. Blood was centrifuged at 1,000 × *g* for 15 min, and a serum was collected. The concentration of FITC-dextran in serum samples was analyzed using a fluorescence spectrophotometer.

### Statistical Analysis

All quantitative data are expressed as mean ± standard error of the mean. The results were analyzed using one-way analysis of variance (ANOVA) with *post hoc* Tukey test or Kruskal–Wallis test with Mann–Whitney *U*-test using Bonferroni correction to adjust the probability. A *P*-value of < 0.05 was considered statistically significant.

## Results

### Pravastatin Attenuates Radiation-Induced Intestinal Injury

To investigate the effects of pravastatin on the intestine, we performed localized irradiation on the abdomen of mice. We exposed the whole abdomens of mice to 13.5 Gy using an Xrad-320, which is designed to deliver localized radiation to experimental animals. We first measured apoptotic cell death in the small intestine using TUNEL assays. Apoptosis is a major pathogenic feature of radiation-induced small intestinal injury, and the degree of apoptosis reflects the severity of enteropathy (Hall and Giaccia, 2012). Widespread apoptosis was detected throughout the crypts 12 h after 13.5 Gy of abdominal irradiation (Figures 1A,C). However, significantly fewer apoptotic cells were observed in the pravastatin-treated irradiated group (Figures 1A,C). We then accessed the therapeutic effects of pravastatin on acute radiation-induced intestinal injury. After irradiation, remarkable crypt destruction with edema, crypt abscess, villi shortening, epithelial cell vacuolization, and inflammatory cell infiltration in lamina propria were observed in the intestine at 3 and 6 days (Figures 1B,D). However, treating irradiated mice with pravastatin significantly rescued crypt damage and villi length compared to that in the IR group (Figures 1B,D). As well as the degree of inflammatory cell infiltration in lamina propria and crypt abscess were reduced. Therefore, pravastatin treatment improves radiation-induced intestinal injury and has anti-apoptotic effects.

The article "Pravastatin Attenuates Acute Radiation-Induced Enteropathy and Improves Epithelial Cell Function" was published in 2018. Journal: Front Pharmacol.

**FIGURE 1:** Pravastatin attenuates radiation-induced intestinal injury. **(A)** TUNEL assay of small intestine tissue from control (Con), irradiated (IR), and pravastatin-treated IR (IR + Prava) mice 12 h after application of 13.5 Gy of abdominal irradiation. Arrows indicate TUNEL-positive cells. Bar = 20 μm. **(B)** H&E-stained intestine tissues harvested from Con, IR, and IR + Prava mice 3 and 6 days after 13.5-Gy irradiation. Bar = 200 μm. **(C)** the number of TUNEL positive cells of small intestinal crypts from Con, IR, and IR + Prava mice 12 h after application of 13.5 Gy of abdominal irradiation. **(D)** Villi lengths in the small intestine from Con, IR, and IR + Prava mice at 3 and 6 days after irradiation. Data are presented as the mean ± standard error of the mean; *n* = 5 mice per group. *^∗^P* < 0.05 compared to the control; *^#^P* < 0.05 compared to the IR group.

### Pravastatin Normalizes Impaired Epithelial Cell Differentiation in the Irradiated Intestine

Stem cells residing in the crypts of Lieberkuhn of the small intestine produce progenitor cells that differentiate into goblet cells, enterocytes, enteroendocrine cells, and Paneth cells (Haegebarth and Clevers, 2009). To identify the effect of pravastatin on epithelial cell differentiation in the small intestine, we performed immunohistochemistry for MUC2, a goblet cell marker, ChgA, a marker of enteroendocrine cells, and Lyz1, a Paneth cell marker, in small intestine tissue. Destruction of both crypts and villi, with a reduction in the number of both goblet and enteroendocrine cells, which also appeared irregular in shape, were depicted in the IR mice (Figures 2A,B). However, the cell showing immunoreactive for MUC2 and ChgA are increased in pravastatin treated IR mice compared to that in the IR mice (Figures 2A,B). Therefore, pravastatin treatment prevented damage to goblet and enteroendocrine cells in the irradiated intestine (Figures 2A,B). Paneth cells produce defensins to protect the small intestine against bacterial entrance. The localization of Paneth cells changed from the bottom of crypt to the tip of the villi, and exhibited abnormal forms, in the intestine of the IR group (Figure 2C). However, normalized Paneth cell location and form were observed in the irradiated intestine of pravastatin-treated IR mice (Figure 2C). Taken together, pravastatin treatment protects against impaired epithelial differentiation induced by radiation exposure.

The article "Pravastatin Attenuates Acute Radiation-Induced Enteropathy and Improves Epithelial Cell Function" was published in 2018. Journal: Front Pharmacol.

**FIGURE 2:** Pravastatin normalizes impaired epithelial cell differentiation in the irradiated intestine. Expression of **(A)** MUC2, **(B)** ChgA, and **(C)** Lyz1 in the intestine tissue of control (Con), irradiated (IR), and pravastatin-treated IR (IR + Prava) mice, as detected by immunohistochemistry. Bar = 100 μm. Data are presented as the mean ± standard error of the mean; *n* = 5 mice per group.

### Pravastatin Enhances Epithelial Cell Proliferation After Radiation-Induced Intestinal Damage

Because pravastatin effectively protected against damage to intestinal epithelial cells, according to the histological analysis, we sought to confirm the effects of pravastatin on intestinal epithelial cells using *in vitro* and *in vivo* systems. We treated InEpC cells, which are human normal intestinal epithelial cells with stem cell properties, with different concentrations of pravastatin (0–10 μM) and examined proliferation. WST-1 assays showed that that cells significantly increased numbers of proliferating cells with pravastatin, in a dose-dependent manner 48 h after radiation exposure (Figure 3A). Next, we investigated radiation-induced cellular senescence in pravastatin-treated, irradiated InEpC cells. As expected, cytochemical senescent phenotype analysis involving SA β-Gal staining showed that most irradiated InEpC cells displayed cellular senescence, whereas the number of SA β-Gal-positive cells was significantly reduced in pravastatin-treated irradiated InEpC cells (Figure 3B).

**FIGURE 3:** Pravastatin enhances epithelial cell proliferation after radiation-induced intestinal damage. **(A)** WST-1 assays and **(B)** SA β-gal staining of control (Con), irradiated (IR), and pravastatin-treated IR (IR + Prava) InEpC cells. *n* = 3 per group. **(C)** Counting of Ki-67-positive cell in the intestine of Con, IR, and IR + Prava mice. Bar = 200 μm. Data are presented as the mean ± standard error of the mean; *n* = 5 mice per group. *^∗^P* < 0.05 compared to the control; *^#^P* < 0.05 compared to the IR group.

The article "Pravastatin Attenuates Acute Radiation-Induced Enteropathy and Improves Epithelial Cell Function" was published in 2018. Journal: Front Pharmacol.

To assess the proliferative activity of epithelial cells in pravastatin-treated irradiated mice, we performed immunohistochemistry for the proliferation marker Ki-67 on intestine tissue specimens. The intestines of the IR mice exhibited few Ki-67-positive cells, whereas those of pravastatin-treated IR mice showed increased Ki-67 positivity in the crypt (Figure 3C). Therefore, pravastatin improves epithelial proliferation after radiation-induced intestinal injury.

### Pravastatin Attenuates Radiation-Induced Oxidative Stress in the Intestinal Epithelial Cells

Oxidative stress, a critical cause of radiation-induced injury, could play a role in altered epithelial proliferation, increased apoptosis, and DNA damage (Jacobson, 1996; Keates et al., 1997; Ding et al., 2007). Thus, we examined whether pravastatin treatment reduces radiation-induced oxidative stress in intestinal epithelial cells. To investigate the effect of pravastatin on mitochondrial superoxide production and cellular ROS damage in epithelial cells after irradiation, we performed MitoSOX and DCF-DA assays using pravastatin-treated irradiated InEpC cells. The number of MitoSOX-positive cells and fluorescence intensity were significantly increased in irradiated InEpC cells (Figure 4A). However, the number of MitoSox-positive cells and fluorescence intensity were remarkably reduced in the pravastatin-treated IR InEpC group compared to that in the IR InEpC group (Figure 4A). We also identified that pravastatin treatment attenuated cellular ROS generation in irradiated InEpC cells through DCF-DA assays (Figure 4B). GSH, a well-known antioxidant, provides important protection against oxidative injury by participation in the cellular system of defense against oxidative damage. GSH levels were significantly increased in the pravastatin-treated IR InEpC group compared to that in the IR InEpC group (Figure 4C). Next, we analyzed oxidative damage in irradiated mice using the ROS-induced DNA damage marker, 8-OHdG (Figure 4D). Whereas 8-OHdG was present in the tip of villi of the normal intestine, expression of 8-OHdG was widespread in epithelial cells of the IR mice (Figure 4D). However, the application of pravastatin limited the expression of 8-OHdG in the irradiated intestine (Figure 4D). Taken together, pravastatin suppresses radiation-induced oxidative damage in intestinal epithelial cells.

**FIGURE 4:** Pravastatin attenuates radiation-induced oxidative stress in intestinal epithelial cells. **(A)** MitoSox Red assay, **(B)** 2′,7′-dichlorofluorescein diacetate (DCF-DA) assay, and **(C)** glutathione (GSH) assay of control (Con), irradiated (IR), and pravastatin-treated IR (IR + Prava) InEpC cells. *n* = 3 per group. **(D)** Immunohistochemistry analysis of 8-OHdG in the small intestine of Con, IR, and IR + Prava mice. Arrows indicate 8-OHdG-positive cells. Bar = 50 μm. Data are presented as the mean ± standard error of the mean; *n* = 5 mice per group. *^∗^P* < 0.05 compared to the control; *^#^P* < 0.05 compared to the IR group.

The article "Pravastatin Attenuates Acute Radiation-Induced Enteropathy and Improves Epithelial Cell Function" was published in 2018. Journal: Front Pharmacol.

### Pravastatin Inhibits the Inflammatory Response During Radiation-Induced Intestinal Enteropathy

Increased ROS production in mammary epithelial cells significantly enhances the expression of inflammatory cytokines and nuclear factor kappa light chain enhancer of activated B cells (NF-κB) activity (Li et al., 2017), and contributes to the inflammatory response (Tüzün et al., 2002; Rezaie et al., 2007; Roessner et al., 2008). Because pravastatin treatment reduced oxidative damage in irradiated epithelial cells, we investigated the anti-inflammatory effects of pravastatin during radiation-induced enteritis. A significant increase in epithelial-derived (pro-)inflammatory cytokines such *as interleukin (IL)-6, IL-1β, and tumor necrosis factor-α (TNF-α)* was observed in irradiated InEpC cells (Figures 5A–C). However, pravastatin treatment attenuated the expression of inflammatory cytokines compared to that in the IR group (Figures 5A–C). We also evaluated the anti-inflammatory effects of pravastatin using intestinal tissue subjected to radiation-induced enteropathy. Increases in MPO, a marker of activated neutrophils, correspond to the severity of inflammation in conditions such as inflammatory bowel disease (IBD) and radiation enteritis (Giriş et al., 2006 Kim et al., 2012). MPO-positive cells were significantly increased in the intestine of the IR mice compared to that in the control mice (Figure 5D). However, pravastatin treatment attenuated MPO-positive cells in the irradiated intestine (Figure 5D). *Il-1β, Tnf-α*, and *matrix metallopeptidase 9* (*Mmp9)* expression was shown to markedly increase during acute radiation-induced intestinal injury and play pivotal roles in inflammation (Shim et al., 2017). Thus, we analyzed mRNA levels of *Il-1β, Tnf-α*, and *Mmp9* in the irradiated intestine by real-time RT-PCR. *Il-1β, Tnf-α*, and *Mmp9* expression significantly increased in the intestine of the IR mice, whereas levels of these inflammatory cytokines and chemokine were decreased in the pravastatin-treated IR mice (Figures 5E–G). Thus, pravastatin treatment inhibits the inflammatory response during radiation-induced enteropathy.

**FIGURE 5:** Pravastatin inhibits the inflammatory response during radiation-induced enteropathy. mRNA levels of **(A)** interleukin (*IL)-6*, **(B)** *IL-1β*, and **(C)** tumor necrosis factor (*TNF)-α* in control (Con), irradiated (IR), and pravastatin-treated IR (IR + Prava) InEpC cells, as determined by real-time RT-PCR. *n* = 3 per group. **(D)** Immunohistochemistry analysis of myeloperoxidase (MPO) and mRNA levels of **(E)** *Il-1β*, **(F)** *Tnf-α*, and **(G)** matrix metallopeptidase (*Mmp)-9* in the intestine of Con, IR, and IR + Prava mice. Arrow indicate MPO-positive cells. Bar = 100 μm. Data are presented as the mean ± standard error of the mean; *n* = 5 mice for each group. *^∗^P* < 0.05 compared to the control; *^#^P* < 0.05 compared to the IR group.

The article "Pravastatin Attenuates Acute Radiation-Induced Enteropathy and Improves Epithelial Cell Function" was published in 2018. Journal: Front Pharmacol.

### Pravastatin Rescues Impaired Intestinal Barrier Function After Radiation Exposure

To determine whether pravastatin treatment after radiation exposure can improve epithelial barrier function, we assessed this property by performing bacterial translocation and FITC-dextran absorption assays. Bacterial translocation to the lymph nodes indicates defects in the intestinal barrier, and we determined that irradiation significantly increased bacterial translocation to mLNs compared to that in control mice (Figure 6A). However, treating irradiated mice with pravastatin inhibited bacterial translocation to the mLNs (Figure 6A). We also performed FITC-dextran absorption assays to analyze the localized permeability of the intestine in the pravastatin-treated mice. The concentration of FITC in the serum was significantly increased in the IR mice compared to that in the control mice (Figure 6B). However, pravastatin treatment decreased FITC levels compared to that in the IR mice (Figure 6B). Tight junctions, which are highly specialized intercellular junctions, are responsible for epithelial barrier functions in the gastrointestinal tract (Turner, 2009). Interestingly, mRNA levels of *Cldn3*, a tight junction molecule, were significantly increased in the pravastatin-treated IR mice compared to those in the IR mice at 6 days (Figure 6C). In addition, we also identified that protein expression of CLDN3 was upregulated in the irradiated intestine with pravastatin treatment (Figure 6D). These results suggested that pravastatin not only attenuates radiation-induced enteropathy but also improves intestinal barrier dysfunction caused by radiation exposure.

**FIGURE 6:** Pravastatin rescues impaired intestinal barrier function induced by radiation exposure. **(A)** The number of colonies from mLNs tissue and **(B)** FITC-dextran absorption assay of control (Con), irradiated (IR), and pravastatin-treated IR (IR + Prava) mice. **(C)** mRNA and **(D)** protein expression of claudin 3 (CLDN3) in the intestinal tissue of Con, IR, and IR + Prava mice. Bar = 100 μm. Data are presented as the mean ± standard error of the mean; *n* = 5 mice per group. *^∗^P* < 0.05 compared to the control; *^#^P* < 0.05 compared to the IR group.

The article "Pravastatin Attenuates Acute Radiation-Induced Enteropathy and Improves Epithelial Cell Function" was published in 2018. Journal: Front Pharmacol.

## Discussion

The gastrointestinal tract is a major site for the generation of pro-oxidants (Bhattacharyya et al., 2014). Radiation exposure also induces the overproduction of ROS and oxidative stress, which results in the progression to apoptosis, necrosis, and senescence in irradiated cells. These forms of cell damage predominantly appeared in the intestinal crypts, and also induced impaired differentiation of intestinal epithelial cells. Differentiated cells in the intestine can be classified into two groups. One type of absorptive cell (enterocyte) and other types of secretory cells (goblet, Paneth, and enteroendocrine cells) comprise the small intestinal epithelium (Noah et al., 2011). Enterocytes, which are the most abundant cell type in the small intestine, function to absorb nutrients apically and export them basally (Noah et al., 2011). Enteroendocrine cells, comprising approximately 1% of the small intestinal epithelium, secrete hormones (Noah et al., 2011). Paneth cells synthesize antibacterial peptides in the lumen and goblet cells produce mucus to protect the intestinal barrier from noxious luminal contents (Noah et al., 2011). We identified increases in epithelial apoptosis and senescence and impaired epithelial cell proliferation with oxidative damage in irradiated InEpC cells and the mouse model of radiation-induced enteritis. Further, radiation-induced epithelial injury progressed to the abnormal differentiation of intestinal epithelial cells.

Pravastatin, an inhibitor of HMG-CoA reductase, is widely used to treat hypercholesterolemia and has been reported to have therapeutic effects in a range of inflammatory conditions (Rosenson, 1999; Nakamura et al., 2006). Statins also show radioprotective effects due to the inhibition of several inflammatory kinases including Rho and Rho-associated protein kinases, which regulate pro-inflammatory and pro-fibrotic stress responses, respectively (Haydont et al., 2007; Holler et al., 2009; Ostrau et al., 2009). Moreover, pravastatin exerts persistent anti-inflammatory and anti-thrombotic effects on irradiated endothelial cells (Gaugler et al., 2005;Holler et al., 2009) and inhibits radiation-induced increases in blood endothelial cell interactions (Gaugler et al., 2005). However, there was previously limited reports of the post-treatment therapeutic effect of pravastatin on irradiated intestinal epithelial cells. In our study, radiation exposure induced mitochondrial superoxide, cellular ROS, and DNA damage, and inhibited antioxidants in epithelial cells. Otherwise, pravastatin reduced radiation-induced oxidative stress to epithelial cells, suppressed cell damage, and improved proliferation in InEpC cells and whole-abdominal irradiated mice. Taken together, the anti-oxidative effects of pravastatin improves radiation-induced enteropathy with concomitant decreases in apoptosis, increases in proliferation, and the normalization of intestinal epithelial cell differentiation.

The article "Pravastatin Attenuates Acute Radiation-Induced Enteropathy and Improves Epithelial Cell Function" was published in 2018. Journal: Front Pharmacol.

Enhanced ROS production is associated with intestinal inflammation and increased levels of (pro-inflammatory) cytokines such as TNF-α, IL-6, and IL-1β through the activation of NF-κB (Morgan and Liu, 2011; Li et al., 2017). In addition, excessive ROS and oxidative stress occur in response to inflammatory cytokines such as IL-1β (Ginnan et al., 2013) and TNF-α (Frey et al., 2002). Necrotic cells and oxidative stress-induced damaged extracellular matrix in turn release various intracellular and extracellular molecules, which trigger inflammatory cascades (Chan, 2012). The critical roles of oxidative stress on intestinal inflammation such as radiation enteritis and IBD have been described. Increased ROS levels in the intestinal mucosa in animal models of intestinal inflammation are known to be correlated with disease severity and progression (Jena et al., 2012). In addition, inhibition of ROS production could provide an important protective and therapeutic effect against intestinal inflammation (Wang et al., 2008; Tahan et al., 2011; Trivedi and Jena, 2013). We identified increases in epithelial-derived inflammatory cytokines such as IL-1β, TNF-α, and IL-6 with oxidative damage in irradiated InEpC cells. In addition, in our mouse model, inflammatory cytokines and neutrophil infiltration were increased in the irradiated group compared to those in control animals. MPO, a heme enzyme released by activated neutrophils, is associated with infiltration into the inflamed mucosa of the damaged area and dysfunction of the intestinal barrier (Krawisz et al., 1984; Zhou and Liu, 2017). The application of pravastatin inhibited the expression of inflammatory cytokines and MPO activity in *in vitro* and *in vivo* model. Therefore, pravastatin displays anti-inflammatory effects with reduced oxidative stress during radiation-induced enteropathy.

As one of the most important functions of the epithelium is separate the inner-body space from the outer environment, disruption of this barrier function can lead to invasion by bacteria or antigens. The term ‘mucosal barrier’ might include the physical barrier function that is maintained by the cell-to-cell junctions between epithelial cells, and also the anti-microbial functions that are mediated by intestinal epithelial cells. Disruption in the assembly of tight junctions or adherens junctions might lead to the development of spontaneous intestinal inflammation (Laukoetter et al., 2007). Moreover, epithelial cell damage induces intestinal barrier dysfunction resulting in bacterial translocation from the lumen to the blood, which can progress to inflammation and endotoxemia (Fukata et al., 2005; Jang et al., 2018). The increased permeability of gastrointestinal epithelial cells after radiation exposure frequently results from the redistribution of tight junctions (Shukla et al., 2016). In this study, we showed that pravastatin treatment restores the damaged intestinal barrier by performing bacterial translocation assays and FITC-Dextran analysis. In addition, CLDN3 expression was increased by pravastatin treatment during radiation enteropathy. We thus demonstrated that pravastatin has a therapeutic effect on intestinal lesions and attenuates radiation-induced epithelial dysfunction by decreasing oxidative stress and inflammatory responses. Therefore, we suggest that pharmacological modulation of epithelial dysfunction could limit intestinal toxicity after irradiation.

The article "Pravastatin Attenuates Acute Radiation-Induced Enteropathy and Improves Epithelial Cell Function" was published in 2018. Journal: Front Pharmacol.

## Author Contributions

HJ, JL, SP, SS, and JM: conceived and designed the experiments. HJ, JL, HM, JK, KK, HK, S-JL, and SS: performed the experiments. HJ, JL, HM, JK, HK, and SS: analyzed the data. SP, W-SJ, and JM: contributes reagents, material, and analysis tools. HJ, JL, SS, and JM: wrote the paper.

## Conflict of Interest Statement

The authors declare that the research was conducted in the absence of any commercial or financial relationships that could be construed as a potential conflict of interest.

## Abbreviations

8-OHdG: 8-hydroxy-2′-deoxyguanosine
ChgA: chromogranin A
CLDN3: claudin 3
Con: control
DCF-DA: 2′,7′-dichlorofluorescein diacetate
FITC: fluorescein isothiocyanate
GSH: glutathione
H&E: hematoxylin and eosin
HMG-CoA: 3-hydroxy-3-methylglutaryl coenzyme A
InEpC: human intestinal epithelial cell line
IL: interleukin
IR: irradiation
IR + Prava: pravastatin-treated IR
Lyz1: lysozyme 1
KIRAMS: Korea Institute of Radiological and Medical Sciences
Muc2: mucin 2
mLNs: mesenteric lymph nodes
Mmp9: matrix metallopeptidase 9
MPO: myeloperoxidase
NF-κB: nuclear factor kappa light chain enhancer of activated B cells
PBS: phosphate-buffered saline
ROS: reactive oxygen species
RT-PCR: reverse transcription-polymerase chain reaction
SA β-gal: senescence-associated β-galactosidase
SPF: specific pathogen-free
TNF-α: tumor necrosis factor-α
TUNEL: terminal deoxynucleotidyl transferase dUTP nick and labeling
WST-1: water-soluble tetrazolium salts
